The article "Screening of candidate genes and fine mapping of drought tolerance quantitative trait loci on chromosome 4 in rice (Oryza sativa L.) under drought stress" was retracted in 2015. Reasons: errors in the cell lines or tissues; errors in the results or conclusions; unreliable results or conclusions.

# Screening of candidate genes and fine mapping of drought tolerance quantitative trait loci on chromosome 4 in rice (*Oryza sativa* L.) under drought stress

**DOI:** 10.1002/ece3.1786

**Published:** 2015-10-15

**Authors:** Yuan‐Yuan Nie, Lin Zhang, Yun‐Hua Wu, Hao‐Jie Liu, Wei‐Wei Mao, Juan Du, Hai‐Lin Xiu, Xiao‐Yu Wu, Xia Li, Yu‐Wei Yan, Guo‐Lan Liu, Hong‐Yan Liu, Song‐Ping Hu

**Affiliations:** ^1^ College of Bioscience and EngineeringJiangxi Agricultural UniversityNanchang330045China; ^2^ Jiangxi Super‐rice Research and Development Center/National Engineering Laboratory for RiceNanchang330200China; ^3^ Department of Plant and Microbial BiologyUC BerkeleyBerkeleyCalifornia94720; ^4^ Shanghai Agrobiological Gene CenterShanghai201106China

**Keywords:** Candidate genes, drought stress, drought tolerance, fine mapping, quantitative trait loci, rice (*Oryza sativa* L.)

## Abstract

Due to severe water resource shortage, genetics of and breeding for DT (drought tolerance) in rice (*Oryza sativa* L.) have become one of the hot research topics. Identification of grain yield QTLs (quantitative trait loci) directly related to the DT trait of rice can provide useful information for breeding new drought‐resistant and water‐saving rice varieties via marker‐assisted selection. A population of 105 advanced BILs (backcross introgression lines) derived from a cross between Zhenshan97B and IRAT109 in Zhenshan97B background were grown under drought stress in a field experiment and phenotypic traits were investigated. The results showed that in the target interval of RM273‐RM255 on chromosome 4, three main‐effect QTLs related to panicle length, panicle number, and spikelet number per panicle were identified (LOD [logarithm of the odds] > 2.0). The panicle length‐related QTL had two loci located in the neighboring intervals of RM17308‐RM17305 and RM17349‐RM17190, which explained 18.80% and 20.42%, respectively, of the phenotypic variation, while the panicle number‐related QTL was identified in the interval of RM1354‐RM17308, explaining 11.47% of the phenotypic variation. As far as the spikelet number per panicle‐related QTL was concerned, it was found to be located in the interval of RM17308‐RM17305, which explained 28.08% of the phenotypic variation. Using the online Plant‐GE query system, a total of 13 matched ESTs (expressed sequence tags) were found in the target region, and of the 13 ESTs, 12 had corresponding predicted genes. For instance, the two ESTs CB096766 and CA765747 were corresponded to the same predicted gene *LOC_Os04g46370*, while the other four ESTs, CA754286, CB000011, CX056247, and CX056240, were corresponded to the same predicted gene *LOC_Os04g46390*.

The article "Screening of candidate genes and fine mapping of drought tolerance quantitative trait loci on chromosome 4 in rice (Oryza sativa L.) under drought stress" was retracted in 2015. Reasons: errors in the cell lines or tissues; errors in the results or conclusions; unreliable results or conclusions.

## Introduction

Drought is one of most serious worldwide problems in agriculture, and rice is the largest water consumer in crops (Luo and Zhang 2001; Gowda et al. 2011; Luo et al. 2011). The development of drought‐tolerant varieties is largely based on the quick and precise screening of germplasm and breeding materials in water‐limited environments, mapping and cloning the DT (drought tolerance) genes, incorporating the gene of high‐yield, good quality, and DT using MAS (marker‐assisted selection) and transgenic technology (Teng et al. 2002; Steele et al. 2007; Cairns et al. 2009; Bernier et al. 2009). DT is a complex trait that is affected by many morphological and physiological factors. Genetic analysis of DT has resulted in the identification of a large number of QTLs (quantitative trait loci) for DT‐related traits in rice, many QTLs for DT‐related traits (e.g., cell membrane stability, osmotic adjustment, yield‐ and root‐related traits) have been identified (reviewed by Bernier et al. 2008, Kamoshitaa et al. 2008). For example, using the same RILs (recombinant inbred lines) but a different drought treatment method, 32 QTLs for grain yield and its component traits (e.g., spikelet fertility, spikelet number per panicle, 1,000‐grain weight, and panicle number) were identified by Zou et al. (2005). Among them, 18 and 14 QTLs were detected under normal irrigation and drought stress conditions, respectively.

Although numerous QTLs for DT‐related traits have been reported using different genetic populations in rice, very few have been confirmed (reviewed by Bernier et al. 2008 and Kamoshitaa et al. 2008). Co‐location or overlapping analysis of DT‐related QTLs obtained from different research groups or populations revealed that only four QTLs intervals for the traits were reproducibly detected (Kamoshitaa et al. 2008). Steele et al. (2006) created NILs (near‐isogenic lines) of rice by marker‐assisted backcrossing for five root trait‐related QTLs and evaluated their root traits in different field experiments; however, only one root‐related QTL was confirmed (Steele et al. 2006).

On this account, we carried out a series of fine mapping and candidate genes' screening on the DT‐related QTLs under the basis of our works more than a decade and acquired also many good results.

A population of 105 advanced BILs (backcross introgression lines) derived from a cross between Zhenshan97B and IRAT109 in the Zhenshan97B background were grown under drought stress in a field experiment and phenotypic traits were investigated. DT QTLs were fine mapped with markers in the target region of RM273‐RM255 on chromosome 4 of rice. Mapping results combined with bioinformatics were used in the analysis of candidate genes within the target region so as to identify DT‐related grain yield QTLs which not only could provide a theoretical basis for cloning of candidate genes of DT QTLs but also facilitate the breeding of new rice varieties for DT through MAS.

The article "Screening of candidate genes and fine mapping of drought tolerance quantitative trait loci on chromosome 4 in rice (Oryza sativa L.) under drought stress" was retracted in 2015. Reasons: errors in the cell lines or tissues; errors in the results or conclusions; unreliable results or conclusions.

## Materials and Methods

### Plant growth and drought treatment

In this study, a population of NILs derived from a cross between Zhenshan97B and IRAT109 in the background of Zhenshan 97B was used. Zhenshan97B is an improved lowland *indica* rice variety widely grown in South China, and IRAT109 is a drought‐resistant upland *japonica* rice variety developed by the West Africa Rice Development Association and derived from IRAT13 × IRAT10.

The BILs population was developed as follows: From a population of RILs (F_9_) derived from a cross between Zhenshan97B and IRAT109, the lines with the target region RM273‐RM255 on chromosome 4 derived from the drought‐resistant parent IRAT109 and the left genetic background derived more from Zhenshan97B were selected to backcross with Zhenshan97B for three generations and followed by selfing for five generations. Finally, a total of 520 BC_3_F_5_ advanced BILs were obtained. Fifty‐seven pairs of insertion/deletion (InDel) and SSR (simple sequence repeat) markers in the target region were utilized in the analyses of the prospect and background of the population, and 105 lines that could cover the target region were chosen to be used in this study.

### Experimental methods

One hundred and five BILs with the target region on chromosome 4 were grown in a DT screening greenhouse in the Zhonggu Base in Shanghai of China. The experiment was conducted with 3 duplications. To make sure that most of the lines were subjected to drought stress at the early stage of panicle initiation (when the growth of rice is most sensitive to soil moisture), the lines were sown at two different times with 15‐days interval. The population lines and the parent Zhenshan 97B were sown on June 15, and the another parent IRAT109 was shown on May 30. The seedlings were transplanted at the same date of July 6. For each BIL, four rows of 18 hills per row were planted. Hill spacing within a row was 18 cm while spacing between rows was 20 cm. Conventional field management and fertilization were applied.

Before drought treatment, water was supplied to keep the soil saturated. Water supply was stopped for drought treatment when the early stage of panicle initiation began, and the rice plants were subjected to drought stress for 2 weeks. The leaf age of Zhenshan97B is 13.8 day in Shanghai, and the early stage of panicle initiation usually begins at the age of 10 leaves. Twenty days after transplanting when the average leaf age of population was 9–10 leaves old and when plant growth and development was observed by panicle dissection, water supply was stopped. Drought treatment and water management were the same as reported previously (Hu et al. 2009). During treatment, soil moisture content was measured by Trime FM‐3 (IMKO Corporation, Ettlingen, Germany) every 3 days to monitor the process of drought development. The drought treatment was conducted for 39 days, and the traits' investigation was stopped.

The article "Screening of candidate genes and fine mapping of drought tolerance quantitative trait loci on chromosome 4 in rice (Oryza sativa L.) under drought stress" was retracted in 2015. Reasons: errors in the cell lines or tissues; errors in the results or conclusions; unreliable results or conclusions.

### Field traits investigation

The traits of the BILs subjected to drought stress at their early stage of panicle initiation were observed, which included those related to the QTLs identified in the target region (RM273‐RM255) on chromosome 4 by our laboratory or others.

Five plants from the middle two rows of each line under drought stress were selected for traits inquiry using the method of Zou et al.(2005). The traits chosen included grain yield and grain yield‐related traits such as panicle length, panicle number, grain number per panicle, 100‐grain weight, spikelet fertility, spikelet density, etc.

### Markers and QTLs detection

Zhenshan97B is a lowland *indica* rice variety while IRAT109 is an upland *japonica* rice variety. Thereby, InDel loci and SSR loci longer than 10 bp in length in the target region of RM273‐RM255 on chromosome 4 were selected for marker design based on the comparison results of genomic sequences in the target region of Nipponbare and 9311. QTLMapper2.0 (Wang et al. 1999) was used for composite interval mapping so as to locate the main‐effect QTLs based on the developed linkage map and using the measured grain yield‐related traits under drought stress as input data. Markers were screened at the *P *<* *0.05 level, and marker intervals with logarithm of the odds (LOD) > 2.0 were considered to contain QTLs.

### Data analysis

ANOVA and phenotypic correlation analysis were carried out using a fixed effect model on S‐Plus for Windows V6.1 (Insightful Corporation 2001).

## Results

### Screening of markers

A total of 96 pairs of InDel and SSR markers were designed, of which 52 pairs expressed polymorphism in both parents. And of these 52, 20 pairs were used in mapping (Table 1).

**Table 1:** Marker primer sequence in target interval of chromosome 4

Primer name	Sense (5′–3′)	Antisense (5′–3′)
RM273	5′GAAGCCGTCGTGAAGTTACC3′	5′GTTTCCTACCTGATCGCGAC3′
RM5503	5′GGGAAGAAGATAGGAGATGG3′	5′CTCTGGGTACACTTCACGAG 3′
RM5714	5′TTATGTTGGTGTCGGATTTC3′	5′CGATACATTAGGGCCAATC3′
RM451	5′GATCCCCTCCGTCAAACAC3′	5′CCCTTCTCCTTTCCTCAACC3′
RM1354	5′CACGTAAATAATACCCGGCG3′	5′AAGGTATCTGTCGTGGTGGG3′
RM17308	5′AGGACTGAGGACGGCGAAGG3′	5′CGAAGAATCCGCGACACTAACG3′
RM17305	5′GAGATCGAAGACGATCGAGATGC3′	5′GGGATTTGTCCAGTACTCCTCTTCC3′
RM17363	5′GGAGCAGGCATCTGATCTAGGG3′	5′CAGTTGGGCAACAGATCCATCC3′
RM17349	5′TAGCTGCTGGATGTTACCACTGC3′	5′ACCATCTATCGCCACATCTCACC3′
RM17190	5′CCCGGAGTTCGTTTGAATCTGC3′	5′CTACCGGTACCTGCACTGAGACG3′
RM6748	5′ATTGGGTTTCTCATATTATG3′	5′CCAACACTCCTAACTAGTTC3′
RM7051	5′CTCGATGAGCTTGGCGTC3′	5′TTCAGTGTTCATCGCCTCTG 3′
RIO4024	5′AGCCACTCACGCTCGCCAC3′	5′GCCCAGCAAACGCACCAAA3′
RIO4026	5′TTCAATGGACAAACACAAAGGT3′	5′GTAGGAGTGACAGAAACGCGAC3′
RIO4032	5′TCGTTGCGGGAGAACATTGC3′	5′TCGTCCACTTACTTCTCGCCG3′
RIO4037	5′ATGAGAGAAATCGCTCGCTGCTG3′	5′GTATAAAAATTGTCCCCATACGC3′
RIO4046	5′CCCAAAAATCTCCGTTTCTCAGG3′	5′CTGCGAATACTTATGGCGTGC3′
RIO4047	5′ACGAGGAGTTGATTTGCGTTGTC3′	5′TTCTCGTCCCTGTATGCTTTTGA3′
RIO4052	5′TGGACCCACCAATTTAAGTGAA3′	5′AACGAGGTGAACCATTAACTCATG3′
RM255	5′TGTTGCGTGTGGAGATGTG3′	5′CGAAACCGCTCAGTTCAAC3′

The article "Screening of candidate genes and fine mapping of drought tolerance quantitative trait loci on chromosome 4 in rice (Oryza sativa L.) under drought stress" was retracted in 2015. Reasons: errors in the cell lines or tissues; errors in the results or conclusions; unreliable results or conclusions.

### Soil moisture changes in the greenhouse

Before drought stress, the highest moisture content and the lowest moisture content of soil in the greenhouse were very close, ranging from 44.1% to 43.1%. However, after drought stress just began, the moisture content was kept at approximately 30% at the highest point while that at the lowest point decreased rapidly. Five days after water supply was stopped, moisture difference between the highest point and the lowest point was 6.5% and increased gradually with time. Two weeks after water supply was stopped, difference between the control (no drought treatment) and drought stress was observed with soil moisture content difference of 15.6%. Thirty‐two days after drought stress, the soil moisture content for the highest point and the lowest point was 31.5% and 9.6%, respectively, with a difference of 21.9% (Fig. 1). The results, therefore, showed that the drought stress treatment was sufficient compared to the control in soil moisture content in the greenhouse. In another word, in the control, sufficient soil water was favorable for rice growth while in the drought stress treatment, insufficient soil moisture content inhibited rice growth.

**Figure 1:** Moisture content in 0‐ to 20‐cm‐depth soil layer during the period of drought treatment and control.

### Trait analysis of the BILs and their parents

Table 2 showed the phenotypic values of the nine traits measured under drought stress and their differences between parents and segregation among the population. ANOVA results showed that except panicle number per plant, the other traits were significantly (*P *<* *0.05 or *P *<* *0.001) different between parents and that the traits differed greatly in the population. The traits had a skewness ranging between −1 and +1, presenting a near‐Gaussian distribution and displaying apparent two‐way transgressive segregation.

The article "Screening of candidate genes and fine mapping of drought tolerance quantitative trait loci on chromosome 4 in rice (Oryza sativa L.) under drought stress" was retracted in 2015. Reasons: errors in the cell lines or tissues; errors in the results or conclusions; unreliable results or conclusions.

**Table 2:** Trait performance of parents and BILs (backcross introgression lines) under drought stress

Traits	Drought stress						
	Zhenshan97B	IRAT109	*F* value^1^	Means of BILs	Range of BILs	Skewness	cv
	Means (means ± errors)						
Grain yield per plant, g	3.34 ± 0.51	9.01 ± 1.57	35.53**	7.19 ± 1.64	2.78~11.62	−0.12	0.23
Panicle number	5.00 ± 1.00	3.67 ± 0.58	4.00	8.15 ± 2.21	4.67~14.33	0.79	0.27
Panicle length, cm	15.40 ± 1.01	22.75 ± 0.26	147.92**	16.84 ± 1.65	12.52~20.02	−0.27	0.10
Spikelet number	47.61 ± 10.31	107.17 ± 13.25	37.76**	71.34 ± 13.99	43.80~99.87	0.06	0.20
Spikelet fertility, %	0.68 ± 0.03	0.76 ± 0.01	16.27*	0.62 ± 0.10	0.32~0.80	−0.57	0.16
100‐grain weight, g	2.13 ± 0.03	3.01 ± 0.20	60.44**	1.94 ± 0.12	1.68~2.20	0.01	0.06
Panicle weight, g	0.69 ± 0.16	2.55 ± 0.88	12.94*	0.92 ± 0.24	0.40~1.41	−0.12	0.26
Grain number	32.63 ± 7.49	80.94 ± 9.83	45.82**	44.58 ± 11.72	19.59~73.01	−0.05	0.26
Spikelet density	3.07 ± 0.50	4.71 ± 0.59	13.38*	4.21 ± 0.55	3.05~5.79	0.30	0.13

^1^ *F* value are the ANOVA results between two parents under drought stress.

**P =* *0.01, *P =* *0.05; **is significant at 0.01 level, *is significant at 0.05 level.

Under drought stress, some traits of the parent Zhenshan97B were significantly lower than that of the parent IRAT109 in grain yield, panicle length, spikelet number per panicle, spikelet fertility, 100‐grain weight, panicle weight, grain number per panicle, and spikelet density; however, its panicle number per plant was slightly higher but not significantly different than that of IRAT109. The average spikelet fertility of the population was lower than that of the low value parent Zhenshan97B, but the average panicle number per plant was higher than that of the high value parent Zhenshan97B, showing that these two traits were of transgressive inheritance. However, the other traits of the population had averages between the two parents.

### Correlation analysis and path analysis of population traits

Tables 3 and 4 showed the results of the correlation analysis and path analysis of grain yield and the other trails under drought stress.

**Table 3:** Correlation coefficients between traits under drought stress

Traits	Grain yield/plant	Panicle number	Panicle length	Spikelet number	Spikelet fertility percentage	100‐grain weight	Panicle weight	Grain number	Spikelet density
Panicle number	0.37**	1.00							
Panicle length	0.31**	−0.50**	1.00						
Spikelet number	0.19	−0.59**	0.83**	1.00					
Spikelet fertility percentage	0.46**	−0.30**	0.17	0.09	1.00				
100‐grain weight	0.19	−0.06	0.32**	0.13	−0.04	1.00			
Panicle weight	0.47**	−0.61**	0.75**	0.74**	0.67**	0.22*	1.00		
Grain number	0.42**	−0.61**	0.72**	0.78**	0.68**	0.07	0.96**	1.00	
Spikelet density	0.06	−0.54**	0.52**	0.91**	0.02	−0.04	0.57**	0.66**	1.00

**P =* *0.01, *P =* *0.05; **is significant at 0.01 level, *is significant at 0.05 level.

The article "Screening of candidate genes and fine mapping of drought tolerance quantitative trait loci on chromosome 4 in rice (Oryza sativa L.) under drought stress" was retracted in 2015. Reasons: errors in the cell lines or tissues; errors in the results or conclusions; unreliable results or conclusions.

**Table 4:** Direct and indirect path coefficient, and phenotypic correlations (*R*) between grain yield (*Y*) and yield components (*X*_*i*_) under drought stress

		X1→Y	X2→Y	X3→Y	X4→Y	X5→Y	X6→Y	X7→Y	X8→Y	*R*_*i*,*y*_
Panicle number	X1→	0.649	−0.326	−0.385	−0.193	−0.037	−0.396	−0.397	−0.348	0.371
Panicle length	X2→	−0.340	0.678	0.562	0.116	0.217	0.511	0.486	0.354	0.314
Spikelet number	X3→	−0.645	0.462	−0.778	−0.069	−0.101	−0.576	−0.606	−0.706	0.188
Spikelet fertility percentage	X4→	0.043	−0.143	0.083	0.483	−0.021	0.321	0.328	0.008	0.465
100‐grain weight	X5→	−0.001	−0.001	0.004	0.002	0.013	0.003	0.001	−0.001	0.189
Panicle weight	X6→	0.214	−0.588	0.727	0.715	0.642	0.965	0.924	0.551	0.472
Grain number	X7→	−0.574	0.366	−0.429	−0.467	−0.407	−0.040	−0.599	−0.394	0.424
Spikelet density	X8→	0.532	−0.434	0.423	0.734	0.013	−0.033	0.462	0.809	0.060

Under drought stress, grain yield per plant was significantly (*P *<* *0.001) and positively correlated with panicle number, panicle length, spikelet fertility, panicle weight, and grain number per panicle with correlation coefficients of 0.37, 0.31, 0.46, 0.47 and 0.42, respectively, indicating that the decrease in rice grain yield under drought stress was caused by the decrease in these traits and that rice grain yield can be indirectly raised by genetically improving these traits. Thereby, these traits can reflect the DT trait of rice to some degree. Nevertheless, gain yield per plant had weak and insignificant correlation with spikelet number per panicle, 100‐grain weight, and spikelet density with correlation coefficients of 0.19, 0.19, and 0.06, respectively.

The results of path analysis showed that under drought stress, the correlation coefficient and the direct path coefficient between spikelet fertility and grain yield were close and at the same direction. On the contrary, the correlation coefficients and the direct path coefficients between spikelet number per panicle or grain number per panicle and grain yield had opposite directions. Panicle weight had the greatest direct effect on grain yield with a direct path coefficient of 0.965. But the correlation coefficient between panicle weight and grain yield was only 0.472. This is because panicle weight also has a great negative effect on grain yield via such traits as panicle length.

### Fine mapping of DT QTLs in the target region

Under drought stress, a main‐effect QTL associated with both panicle length and spikelet number per panicle was fine mapped in the target interval RM17308‐RM17305 on chromosome 4 with additive effect of −0.72 cm and −5.98, explaining 18.80% and 28.08% of the phenotypic variations, respectively. Another QTL associated with panicle length was mapped in the target region RM17349‐RM17190 with additive effect and contribution rate of −0.75 cm and 20.42% (Table 5), respectively. It was found that additive effect alleles of q*PL*‐*4b* and q*SN*‐*4* came from the parent IRAT109. The QTL controlling panicle number was located in the region RM1354‐RM17308 with an additive effect of 0.78, explaining 11.47% of the phenotypic variation. Its additive effect allele came from the parent Zhenshan97B. The above two regions were neighbors on chromosome 4 (Fig. 2).

The article "Screening of candidate genes and fine mapping of drought tolerance quantitative trait loci on chromosome 4 in rice (Oryza sativa L.) under drought stress" was retracted in 2015. Reasons: errors in the cell lines or tissues; errors in the results or conclusions; unreliable results or conclusions.

**Table 5:** Quantitative trait loci fine mapping of target regions under drought conditions in chromosome 4

Trait	Loci	Interval	Logarithm of the odds	Additive	*H* ^2^, %
Panicle length	*qPL‐4a*	RM17308‐RM17305	4.23	−0.72	18.80
Panicle length	*qPL‐4b*	RM17349‐RM17190	2.62	−0.75	20.42
Panicle number	*qPN‐4*	RM1354‐RM17308	2.67	0.78	11.47
Spikelet number	*qSN‐4*	RM17308‐RM17305	7.71	−5.98	28.08

**Figure 2:** Quantitative trait loci fine mapping of target regions under drought conditions in chromosome 4.

### QTL effect analysis

QTLs associated with panicle length, panicle number, and spikelet number per panicle were identified in the target region RM1354‐RM17305 under drought stress. The population was grouped based on marker genotype as shown in Table 6 with phenotype information.

**Table 6:** Phenotype data of different genotype for target region on chromosome 4

Genotype	Yield/plant, g	Panicle number	Panicle length, cm	Spikelet number	Spikelet fertility, %	100‐grain weight, g	Panicle weight, g	Grain number	Spikelet density
++/++	7.47 ± 1.48	7.52 ± 1.99*	17.87 ± 1.22**	79.63 ± 11.84**	0.63 ± 0.10	1.99 ± 0.11	1.03 ± 0.22*	49.99 ± 11.01*	4.44 ± 0.47
− −/− −	7.38 ± 1.25	8.59 ± 2.27*	16.31 ± 1.46**	68.93 ± 10.97**	0.62 ± 0.11	1.94 ± 0.13	0.90 ± 0.23*	43.21 ± 11.41*	4.21 ± 0.45

++/++ means the genetic background from IRAT109; − −/− − means the genetic background from Zhenshan 97B.

**P =* *0.01,*P =* *0.05; **is significant at 0.01 level, *is significant at 0.05 level.

As shown from Table 6, there were no significant differences in grain yield per plant, spikelet fertility, 100‐grain yield, and spikelet density between genotypes. The genotypes with alleles coming from IRAT109 had significantly higher panicle length, spikelet number per panicle, panicle weight, and grain number per panicle but significantly lower panicle number than the genotypes with alleles coming from Zhenshan97B. Therefore, this could well explain the fact that QTLs associated with panicle length, panicle number, and spikelet number per panicle were identified in the target region RM1354‐M17305.

The article "Screening of candidate genes and fine mapping of drought tolerance quantitative trait loci on chromosome 4 in rice (Oryza sativa L.) under drought stress" was retracted in 2015. Reasons: errors in the cell lines or tissues; errors in the results or conclusions; unreliable results or conclusions.

### Candidate gene analysis in the target region

The target region RM273‐RM255 on chromosome 4 was narrowed down to the hot region RM17308‐RM17305 via marker for candidate gene analysis using the online Plant‐GE query system (Zeng et al. 2007). The physical position of the hot region on chromosome was 27,444,462‐27,608,347. A total of 13 matched ESTs (expressed sequence tags) were found in the target region and of the 13 ESTs, 12 had corresponding predicted genes. For example, the two ESTs CB096766 and CA765747 were corresponded to the same predicted gene *LOC_Os04g46370* which represented the l‐asparaginase precursor protein, and other four ESTs, CA754286, CB000011, CX056247, and CX056240, were corresponded to the same predicted gene *LOC_Os04g46390* which stood for the chaperone protein DnaJ.

Table 7 showed the functions of the genes. The probable functions of other candidate genes were as follows: CA762215 was parallelism to the gene *LOC_Os04g46310* which would express the HEAT repeat family protein; CA760699 was corresponded to the gene *LOC_Os04g46350* which represented the homeobox‐associated leucine zipper; BE040653 was matched to the gene *LOC_Os04g46460* which might generate amino acid kinase; CA764601 was homologous with the gene *LOC_Os04g46480* which would produce the carotenoid cleavage dioxygenase 7 or chloroplast precursor; CA756239 was corresponded to the gene *LOC_Os04g46530* which could form the retrotransposon protein and the last one is the CA759049 which was matched to the gene *LOC_Os04g46560* with the function of expressing lactate or malate dehydrogenase.

**Table 7:** Putative genes with transcript factor domain

Expressed sequence tags Acc.	Putative gene	Location	Putative function description
CA762215	*LOC_Os04g46310*	27444462–27460087 bp	HEAT repeat family protein, putative, expressed
CA760699	*LOC_Os04g46350*	27479717–27477579 bp	Homeobox‐associated leucine zipper, putative, expressed
CB096766	*LOC_Os04g46370*	27498017–27494465 bp	l‐asparaginase precursor protein, putative, expressed
CA765747	*LOC_Os04g46370*	27498017–27494465 bp	l‐asparaginase precursor protein, putative, expressed
CA754286	*LOC_Os04g46390*	27505490–27510048 bp	Chaperone protein dnaJ, putative, expressed
CB000011	*LOC_Os04g46390*	27505490–27510048 bp	Chaperone protein dnaJ, putative, expressed
CX056247	*LOC_Os04g46390*	27505490–27510048 bp	Chaperone protein dnaJ, putative, expressed
CX056240	*LOC_Os04g46390*	27505490–27510048 bp	Chaperone protein dnaJ, putative, expressed
CA763901	*/*	/	/
BE040653	*LOC_Os04g46460*	27563230–27564681 bp	Amino acid kinase, putative, expressed
CA764601	*LOC_Os04g46480*	27567824–27570926 bp	Carotenoid cleavage dioxygenase 7, chloroplast precursor, putative, expressed
CA756239	*LOC_Os04g46530*	27596150–27592239 bp	Retrotransposon protein, putative, unclassified, expressed
CA759049	*LOC_Os04g46560*	27605166–27608347 bp	Lactate/malate dehydrogenase, putative, expressed

http://rice.plantbiology.msu.edu/cgi-bin/gbrowse/rice/.

The article "Screening of candidate genes and fine mapping of drought tolerance quantitative trait loci on chromosome 4 in rice (Oryza sativa L.) under drought stress" was retracted in 2015. Reasons: errors in the cell lines or tissues; errors in the results or conclusions; unreliable results or conclusions.

So the candidate genes of hot region RM17308‐RM17305 in the target region RM273‐RM255 on chromosome 4 were extensive and various, and their functions referred to heat‐shock protein, leucine zipper, chaperone or retrotransposon protein, and some enzymic formation such as Asparaginase, amino acid kinase, and partial dehydrogenase, etc.

## Discussion

### Tangibility of QTL for DT‐related traits

Many important agronomic traits, especially stress resistance, have a complex genetic basis and are controlled by a large number of QTLs. To understand the genetic and molecular mechanisms controlling such traits, QTLs analyses have been undertaken in many plant species. However, many environmental factors affect the accuracy and repeatability of phenotyping of complex traits. Although some indices for DT, including root traits, leaf rolling, water‐using efficiency, osmotic adjustment, yield, and relative yield traits, have been used to detect DT‐related QTLs, the stability of such QTLs was very low under different conditions. For example, of the 36 genomic regions reported to harbor root trait‐related QTLs (Yue et al.^2006^), only four had positional correspondence with previously identified QTLs for root or other drought avoidance‐related traits (Courtois et al. 2009; Yonemaru et al. 2010).

Because of the low reproducibility of detecting DT‐related QTLs using RIL populations, the tangibility of these QTLs were questionable. Previously, four intervals carrying QTLs for root traits were targeted for generating introgression lines, but only one line with one of these targeting QTLs showed significantly increased root length (Steele et al.^2006^). In this study, NILs were developed to examine 8 QTLs identified previously (Zou et al. 2005). Four NILs of targeting GY‐related QTLs showed significantly phenotypic differences in the corresponding traits.

In recent years, researchers around the world have mapped some main‐effect QTLs influencing the physiological and grain yield traits of rice under irrigation and drought stress conditions using different mapping populations. A comparison between the QTLs identified in this study and those reported in the literature showed that both differences and similarities existed in these QTLs identified in different environments using the same population. The main‐effect QTLs associated with panicle number, tiller number, leaf water potential, canopy temperature, stem base width, and thousand kernel weight were mapped in the 30‐kb region RIO02002‐RM02002 narrowed down from the target region RM561‐RM341 on chromosome 2 via molecular marker by Nie et al. (2012) using the advanced BILs population. Panicle length–associated QTLs, panicle number–associated QTLs, and spikelet number per panicle–associated QTLs were mapped in RM17169‐RM17183, RM5320‐RM17355, and RM5320‐RM17355, respectively, within the target region RM273‐RM255 on chromosome 4 via molecular marker by Liu (2007). The fact that the three QTLs were repeatedly identified in this study confirmed the real existence of these QTLs in the region and the region was further narrowed down in the study.

The article "Screening of candidate genes and fine mapping of drought tolerance quantitative trait loci on chromosome 4 in rice (Oryza sativa L.) under drought stress" was retracted in 2015. Reasons: errors in the cell lines or tissues; errors in the results or conclusions; unreliable results or conclusions.

### Potential exploitation of yield and DT improvement in rice

It is noted that in the important region RM17308‐RM17305 where QTLs associated with traits such as panicle length and spikelet number per panicle were detected in this study, grain yield‐related QTLs were also detected in other populations under drought stress. Candidate gene analysis of the hot region RM17308‐RM17305 showed that the EST CA760699‐corresponding gene *LOC_Os04g46350* was associated with stress resistance of rice. By constructing NILs of the target region on chromosome 4, Ding et al. (2011) managed to fine map the main‐effect *qFSR4* controlling root volume, flag leaf width, and spikelet number per panicle in the neighboring regions of FSR‐75 and FSR‐78 and successfully clone the related gene *NAL1*. Comparing the candidate gene from this study and the cloned DT gene *NAL1*, we found that they were located neighboring to each other in the target region. In the DH (double haploid) population constructed from CT9993 with a upland rice background and lowland *indica* variety IR62266, QTLs associated with root traits, spikelet number, and biological yield were mapped in this region (Zhang et al. 2001; Klueva and Chamareck 2004; Lanceras et al. 2004). Comparison of the mapping results in different environments demonstrated that DT QTLs can be repeatedly detected in the same locus using different materials and different detection methods, showing that these QTLs may be of significance in MAS.

## Conclusions

In conclusion, we have obtained candidate genes which were fine mapped to the some important DT QTLs on the chromosomes 4 of the rice using a population of advanced BILs through CIM methods and the online Plant‐GE query system in this study. Three main‐effect QTLs related to panicle length, panicle number, and spikelet number per panicle were identified. Using the online Plant‐GE query system, a total of 13 matched ESTs were found in the target region, and of the 13 ESTs, 12 had corresponding predicted genes.

The article "Screening of candidate genes and fine mapping of drought tolerance quantitative trait loci on chromosome 4 in rice (Oryza sativa L.) under drought stress" was retracted in 2015. Reasons: errors in the cell lines or tissues; errors in the results or conclusions; unreliable results or conclusions.

## Data Accessibility

The data of candidate genes analysis were used the online Plant‐GE query system, you may log on the address: http://rice.plantbiology.msu.edu/cgi-bin/gbrowse/rice/.

## Conflict of Interest

The authors declare that they have no conflict of interests.

## References

[ece31786-bib-0001] Bernier, J. , A. Kumar , R. Serraj , D. Spaner , and G. N. Atlin . 2008 Breeding upland rice for drought resistance. J. Sci. Food Agric. 88:927–939.

[ece31786-bib-0002] Bernier, J. , R. Serraj , A. Kumar , R. Venuprasad , S. Impa , V. R. Gowda , et al. 2009 The large‐effect drought‐resistance QTL *qtl12.1* increases water uptake in upland rice. Field. Crop. Res. 110:139–146.

[ece31786-bib-0003] Cairns, J. E. , A. Audebert , C. E. Mullins , and A. H. Price . 2009 Mapping quantitative trait loci associated with root growth in upland rice (*Oryza sativa* L.) exposed to soil water‐deficit in fields with contrasting soil properties. Field. Crop. Res. 114:108–118.

[ece31786-bib-0004] Courtois, B. , N. Ahmadi , F. Khowaja , A. H. Price , J. F. Rami , J. Frouin , et al. 2009 Rice root genetic architecture: meta‐analysis from a drought QTL database. Rice 2:115–128.

[ece31786-bib-0005] Ding, X. P. , X. K. Li , and L. Z. Xiong . 2011 Evaluation of near‐isogenic lines for drought resistance QTL and fine mapping of a locus affecting flag leaf width, spikelet number, and root volume in rice. Theor. Appl. Genet. 123:815–826.2168149010.1007/s00122-011-1629-1

[ece31786-bib-0006] Gowda, V. R. , A. Henry , A. Yamauchi , H. E. Shashidhar , and R. Serraj . 2011 Root biology and genetic improvement for drought avoidance in rice. Field. Crop. Res. 122:1–13.

[ece31786-bib-0007] Hu, S. P. , Y. Zhou , L. Zhang , X. D. Zhu , L. Li , L. J. Luo , et al. 2009 Correlation and quantitative trait loci analyses of total chlorophyll content and photosynthetic rate of rice (*Oryza sativa*) under water stress and well‐watered conditions. J. Integr. Plant Biol. 51:879–888.1972324710.1111/j.1744-7909.2009.00846.x

[ece31786-bib-0008] Insightful Corporation 2001 S‐plus 6 for windows, user's guide, Insightful Corporation, Seattle, WA.

[ece31786-bib-0009] Kamoshitaa, A. , R. C. Babub , N. M. Boopathib , and S. Fukaic . 2008 Phenotypic and genotypic analysis of drought‐resistance traits for development of rice cultivars adapted to rainfed environments. Field. Crop. Res. 109:1–23.

[ece31786-bib-0010] Klueva, N. , and V. Chamareck . 2004 Saturation mapping of QTL regions and identification of putative candidate genes for drought tolerance in rice. Mol. Gen. Genet. 272:35–46.10.1007/s00438-004-1025-515221451

[ece31786-bib-0012] Lanceras, J. C. , G. Pantuwan , B. Jongdee , and T. Toojinda . 2004 Quantitative trait loci associated with drought tolerance at reproductive stage in rice. Plant Physiol. 135:384–399.1512202910.1104/pp.103.035527PMC429392

[ece31786-bib-0013] Liu, G. L. 2007 Mapping and evaluation of drought resistant traits of cultivated rice and its applications on rice breeding. Doctoral diss. Huazhong Agricultural University, Wuhan, China Pp. 31–95.

[ece31786-bib-0014] Luo, L. J. , and Q. F. Zhang . 2001 The status and strategy on drought resistance of rice (*Oryza sativa* L.). Chin. J. Rice Sci. 15:209–214.

[ece31786-bib-0015] Luo, L. J. , H. W. Mei , X. Q. Yu , H. Y. Liu , and F. J. Feng . 2011 Water‐saving and drought resistance rice and its development strategy (in Chinese). Chin. Sci. Bull. (Chinese Ver.) 56:804–811.

[ece31786-bib-0016] Nie, Y. Y. , G. H. Zou , Y. Li , G. L. Liu , Y. H. Cai , L. H. Mao , et al. 2012 Fine mapping of drought resistance QTL on chromosome 2 in rice. Acta Agron. Sin. 3:988–995.

[ece31786-bib-0017] Steele, K. A. , A. H. Price , H. E. Shashidhar , and J. R. Witcombe . 2006 Marker‐assisted selection to introgress rice QTLs controlling root traits into an Indian upland rice variety. Theor. Appl. Genet. 112:208–221.1620850310.1007/s00122-005-0110-4

[ece31786-bib-0018] Steele, K. A. , D. S. Virk , R. Kumar , S. C. Prasad , and J. R. Witcombe . 2007 Field evaluation of upland rice lines selected for QTLs controlling root traits. Field. Crop. Res. 101:180–186.

[ece31786-bib-0019] Teng, S. , Q. Qian , D. L. Zeng , G. S. Guo , B. K. Teng , D. N. Huang , et al. 2002 Analysis of gene loci and epistasis for drought tolerance in seedling stage of rice (*Oryza sativa* L.). Acta Genet. Sin. 29:235–240.12182078

[ece31786-bib-0020] Wang, D. L. , J. Zhu , Z. K. Li , and A. H. Paterson . 1999 Mapping QTLs with epistatic effects and QTL×environment interactions by mixed linear model approaches. Theor. Appl. Genet. 99:1255–1264.

[ece31786-bib-0021] Yonemaru, J. , T. Yamamoto , S. Fukuoka , Y. Uga , K. Hori , and M. Yano . 2010 Q‐TARO: QTL annotation rice online database. Rice 3:194–203.

[ece31786-bib-0022] Yue, B. , W. Y. Xue , L. Z. Xiong , X. Q. Yu , L. J. Luo , K. H. Cui , et al. 2006 Genetic basis of drought resistance at reproductive stage in rice: separation of drought tolerance from drought avoidance. Genetics 172:1213–1228.1627241910.1534/genetics.105.045062PMC1456219

[ece31786-bib-0023] Zeng, H. , L. Luo , W. Zhang , J. Zhou , Z. Li , H. Liu , et al. 2007 Plant QTL‐GE: a database system for identifying candidate genes in rice and Arabidopsis by gene expression and QTL information. Nucleic Acids Res. 35:879–882.10.1093/nar/gkl814PMC166973517142239

[ece31786-bib-0024] Zhang, J. , H. G. Zheng , A. Aarti , G. Pantuwan , T. T. Nguyen , J. N. Tripathy , et al. 2001 Locating genomic regions associated with components of drought resistance in rice: comparative mapping within and across species. Theor. Appl. Genet. 103:19–29.

[ece31786-bib-0025] Zou, G. H. , H. W. Mei , H. Y. Liu , G. L. Liu , S. P. Hu , X. Q. Yu , et al. 2005 Grain yield responses to moisture regimes in a rice population: association among traits and genetic markers. Theor. Appl. Genet. 112:106–113.1623116110.1007/s00122-005-0111-3

